# An 11-year trend of rubella incidence cases reported in the measles case-based surveillance system, Ghana

**DOI:** 10.11604/pamj.2021.39.132.23297

**Published:** 2021-06-15

**Authors:** Anthony Zunuo Dongdem, Elizabeth Alhassan, David Opare, Gifty Boateng, George Bonsu, Kwame Amponsa-Achiano, Badu Sarkodie, Emmanuel Dzotsi, Michael Adjabeng, Seth Afagbedzi, Yakubu Alhassan, Kofi Agyabeng, Franklin Asiedu-Bekoe

**Affiliations:** 1 Department of Epidemiology and Biostatistics, School of Public Health, University of Health and Allied Sciences, Ho, Ghana,; 2 Disease Surveillance Department, Ghana Health Service, Accra, Ghana,; 3 National Public Health and Reference Laboratory, Ghana Health Service, Accra, Ghana,; 4 Expanded Programme on Immunization, Ghana Health Service, Accra, Ghana,; 5 Public Health Division, Ghana Health Service, Accra, Ghana,; 6 Oti Regional Health Directorate, Ghana Health Service, Dambai, Ghana,; 7 World Health Organization, Country Office, Accra, Ghana,; 8 Department of Biostatistics, School of Public Health, University of Ghana, Legon, Accra, Ghana

**Keywords:** Rubella, Ghana, incidence, surveillance, trend

## Abstract

**Introduction:**

rubella is vaccine-preventable and vaccination is the most cost-effective approach to control the disease and avoid the management of congenital rubella syndrome cases. Ghana introduced the rubella vaccine into the routine immunization program in 2013. Since then there have not been any evaluation of the epidemiology of rubella. We determined the disease trends and the population demographics of rubella cases, in the Ghana national measles case-based surveillance system.

**Methods:**

we reviewed the measles case-based surveillance data from 2007 to 2017. Descriptive data statistics was done and expressed as frequencies and proportions. Chi-square test was used to establish associations.

**Results:**

a total of 11,483 suspected cases for measles received and tested for measles IgM antibodies and 1,137(12.98%) confirmed positive for the period. Of these 10,077 were negative and 250 indeterminate for measles and tested for rubella and 2,090 (20.23%) confirmed positive for rubella IgM antibodies. More females (21.45%) were affected than males (19.48%). Majority of the confirmed positives were recorded in the urban areas. Children aged 15 years or less were mostly affected. There was a statistical difference between incidence cases and sex (χ2=6.03, p-value = 0.014), or age (χ2=283.56, p-value < 0.001) or area (χ2= 6.17, p-value = 0.013). Most infections occurred during the dry season.

**Conclusion:**

children less than 15 years were mostly affected with majority being females. The highest incidence of cases was before the rains and occurred mostly in urban areas. The incidence of cases has declined significantly with the introduction of the rubella vaccine.

## Introduction

Rubella is often an unrecognized disease that affects mostly children. It is cause by the rubella virus and is transmitted by inhalation of infective droplets. Incubation period of the disease is from 12 to 23 days (average of 18 days) and the contagious period is from one week before to one week after the onset of rash. Rubella infections are often unrecognized; of concern is the teratogenic effect of the virus during pregnancy which is characterized by multiple birth defects known as congenital rubella syndrome (CRS). These malformations were first observed in 1941 after an outbreak in Australia [1]. Common among these birth defects are ocular, hearing impairment, heart defects, microcephaly, developmental delay, mental retardation, bone alterations, autism and damage to the liver and spleen [2,3]. Although the burden of CRS is not well documented in many countries, more than 100,000 babies with congenital rubella syndrome (CRS) were estimated to be born worldwide in 2010 [2]. In Ghana, an estimated ratio of 8 cases of CRS per 10,000 live births per year occurs [4]. Exposure to rubella is high in the population with 92.6% prevalence in pregnant women in Ghana [4]. Among measles suspected cases that tested negative, up to 40% are positive for rubella because of the similarities in symptoms presentation [5]. Despite the endemicity of rubella and the reported CRS cases in Ghana no specific intervention was put in place until in September 2013 when the combined measles and rubella vaccine was introduced to protect against these diseases. Since then there have not been any systematic evaluation of the incidences of rubella. In order to describe the current changes in the epidemiology of rubella, a population-based incidence study is necessary. The aim of this study therefore is to describe the current disease trends and the population demographics of rubella cases identified through the Ghana national measles case-based surveillance system from 2007 to 2017.

## Methods

**Study design and study site:** we carried out a retrospective data analysis of rubella cases in the national measles case-based surveillance from January 2007 to December 2017. The data was collected at the Disease Surveillance Department (DSD) of the Ghana Health Service, Accra. A suspected case of measles was defined according to the WHO guidelines as: any person with fever and maculopapular (non-vesicular) generalized rash and cough, coryza or conjunctivitis (red eyes) or any person in whom a clinician suspects measles [6]. A confirmed measles case was classified as either laboratory-confirmed, epidemiologically linked or clinically compatible [6].

**Data collection:** the disease control officers completed a case investigation form for each case at the health facility level to collect data on the age, sex, vaccination status, district or village of residence, date of onset and the laboratory results on measles or rubella Immunoglobulin M (IgM), etc. The serum samples are collected within 30 days of onset of the rash and transported to the National Public Health and Reference Laboratory (NPHRL) an accredited laboratory for testing measles and rubella. A case was laboratory confirmed if measles IgM antibodies were detected using the indirect enzyme-linked immunosorbent assay kit. Those with undetectable levels of IgM antibodies were negative or equivocal/indeterminate. The confirmed negatives or equivocal samples were tested for rubella IgM antibodies. The case investigation data together with the laboratory results were entered into the measles case-based surveillance system using the Epi info software.

**Data analysis:** the data obtained was exported into Microsoft Excel, cleaned and analyzed in STATA software version 15 using age, sex, date of onset, area or location, and laboratory IgM results for measles and rubella. Graphs were generated using Microsoft Excel 2013. The demographic categorical data (e.g sex) were presented in summary tables of counts and percentages. For demographic continuous data (e.g. age), summary tables of means, standard deviations were presented. Chi-square test was used to establish associations between demographic data and various outcome variables. All statistical tests were declared significant for p-value < 0.05.

**Ethical issues:** permission to use the national measles surveillance data for the study was obtained from the Head of the National Disease Surveillance Department, Ghana Health Service. Confidentially was maintained by excluding all identifying information such as names, contact information or address that could be linked to the subject from the analysis. The data was stored on a computer and only accessible to the researchers.

## Results

A total of 12,818 suspected cases of measles were reported from all the districts in Ghana from January 2007 to December 2017 to the DSD. The mean age of the cases was 6.28 ± 7.38 years. Among the suspected cases 52.63% (5,435) were males and 46.09% (4,760) females. However, a higher proportion of rubella cases were confirmed among the females (21.45%) than among the males (19.48%) and was found to be statistically significant (χ^2^ = 6.03, p-value = 0.014) (Table 1). Out of the total of the suspected measles cases, 11,483 were tested and 1,137 (12.98%) confirmed positive for measles IgM antibodies. Of the 10,077 cases that tested negative and 250 that were indeterminate for measles, 2,090 (20.23%) of them tested positive for rubella IgM antibodies. Among the negative and indeterminate cases tested for rubella, 19.50% (1131 out of 5800) of those in the rural areas tested positive for rubella whiles 21.50% (942 out of 4381) of those originated from the urban areas tested positive. The difference in incidence of cases in the rural and urban areas was found to be statistically significant (χ^2^ = 6.17, p-value = 0.013) (Table 2).

**Table 1:** demographic characteristics

Variable	Frequency (%)	Confirmed positive (%)	Chi-square	P-value
**Age (mean ± SD)**	6.28 ± 7.38		283.56	˂0.001
˂5 years	4,601	528(11.48)		
5 - 10 years	2,470	626(25.34)		
11 - 15 years	857	229(26.72)		
16 - 20 years	267	60(22.47)		
˃ 20 years	354	44(12.43)		
**Sex**			6.03	0.014
Female	4,760(46.09)	1021(21.45)		
Male	5,435(52.63)	1059(19.48)		
Missing	132(1.28)			
**Area**			6.17	0.013
Rural	5,800	1131(19.50)		
Urban	4,381	942(21.50)		
**Measles cases (N=12,818)**				
Positive	1,137			
Negative	10,077			
Indeterminate	250			
Pending	1,335			
Missing	19			
**Rubella cases (N=10,327)**				
Positive	2,090			
Negative	6,591			
Indeterminate	379			
Pending	1,157			
Missing	110			

**Table 2:** distribution of rubella cases by area from 2007 to 2017

	Rural		Urban	
Year	Total suspected cases	Confirmed positive (%)	Total suspected cases	Confirmed positive (%)
2007	285	76(26.67)	286	97(33.92)
2008	504	190(37.70)	684	265(38.74)
2009	279	85(30.47)	255	47(18.43)
2010	347	90(25.94)	274	70(25.55)
2011	909	341(37.51)	713	251(35.2)
2012	670	200(29.85)	451	128(28.38)
2013	471	106(22.51)	288	60(20.83)
2014	574	25(4.36)	342	13(3.80)
2015	579	8(1.38)	422	4(0.95)
2016	504	7(1.39)	310	4(1.29)
2017	678	3(0.44)	356	3(0.84)
**Total**	**5800**	**1131(19.50)**	**4381**	**942(21.50)**

Among the measles cases for the period, peak incidences occurred in 2012 and 2013 when 289 and 319 cases respectively were confirmed, followed by a sharp decline to 23 cases in 2015 where it remained relatively stable till 2017. On the other hand, rubella confirmed cases recorded its peak incidences in 2008 and 2011 when 459 and 596 cases were respectively recorded. In 2013, 166 cases were recorded and the incidence declined drastically to 12 cases in 2015 and 6 cases in 2017 (Figure 1). The age distribution for rubella showed majority of the rubella cases to occur in the age group 5 to 10 years followed by those under 5 years and the 11 to 15 year group (Figure 2). The differences observed in the age groups were significant (χ^2^ =283.56, p-value < 0.001). A seasonal pattern was observed among the confirmed cases of rubella peaking in February and March. The incidence remained low from August and October as shown in Figure 3. The peak period coincides with the late harmattan (February to April) and the beginning of the rainy season in most parts of the country.

**Figure 1:** trend of confirmed positive measles and rubella cases from 2007 to 2017

**Figure 2:** trend of rubella cases by age group from 2007 to 2017

**Figure 3:** monthly trend of confirmed positive rubella cases by years

## Discussion

The measles surveillance system enabled the detection of the rubella trends in Ghana. In the present analysis conducted, the incidence of rubella cases among the suspected measles cases in the past has been high with the highest peak observed in 2011. The measles cases on the other hand have been relatively lower than the rubella incidences because there have been a vaccination programme since the early 1980s, with Supplementary Immunization activities (SIAs) to develop immunity for those children who fail to induce immunity in response to the first dose. This is not the case with rubella, although the disease is also prevalent. The rubella vaccine was only introduced in September 2013. Since this intervention there have been a drastic decline in the incidence of rubella cases reaching the lowest in 2017. This decline in incidence may be attributed to the introduction of the rubella vaccine which might have conferred protection in the vulnerable populations in most of the communities in the country. It is also observed that the peak incidences of measles and rubella did not coincide as demonstrated by Chimhuya, Manangazira [7] in a similar study in Zimbabwe. This can be explained to occur because of the low incidence of the measles cases which have made the identification of the true measles among suspected cases low by the case definition. However if the measles incidence was high, the clinical case definition would have accurately performed well in identifying measles cases [8]. Thus, if the incidence of measles was low the measles-like rash of the cases detected would be due to rubella. It is also known that up to 50% of persons infected with rubella do not present with rash [9,10]. The rubella rash is not easily recognized on the black skin and may be overlooked [7]. This conversely would have impacted on the CRS cases in Ghana over the years. These suggest that the burden of the rubella cases depicted in the past years may be more than reported and thus was necessary for the rubella vaccine inclusion. As rubella and measles are in the elimination phase, there is the need to adopt a more sensitive case definition that will allow inclusion of all cases for laboratory confirmation. For instance, the Pan American Health Organization for rubella surveillance adopted a new case definition as the region moved towards an elimination target in which a case of rubella was defined as that suspected by a health worker to be rubella [11]. The European Centre for Disease Prevention and Control also adopted a modified definition, namely, any person with sudden onset of generalized maculopapular rash and at least one of the following: cervical adenopathy, sub occipital adenopathy, post auricular adenopathy, arthralgia or arthritis [12]. Therefore, in the elimination phase of rubella, a modified case definition will need to be considered so as to improve on rubella case detection.

Climatic conditions and pattern of human aggregates are known predictors of the seasonal variation of rubella infection [13]. Our study showed a seasonal pattern of rubella cases for the period. It was observed that most of the rubella cases peaked in February and March, a period that coincides with the late hot dry harmattan season and before the beginning of rainy season in most parts of the country in April. Our findings is in consonance with that observed by Chimhuya, Manangazira [7] and Getahun, Beyene [14], who demonstrated high incidence of rubella cases during the hot dry season respectively in Zimbabwe and Ethiopia. Similar variations were also found in the United States and the temperate countries where rubella cases peaked during winter and spring before the introduction of the rubella vaccine [10]. In many other high income countries including England, Wales, Peru, school-driven aggregation have been attributed to the seasonal peaks, such that transmission increases during the school terms and the vice versa [15-17].

In terms of geographical location our study revealed a significantly higher number of rubella cases in the urban areas than the rural areas. This agrees with the findings of Mitiku, Bedada [18] in Ethiopia that reported higher number of positives cases in urban compared to rural settings but contrasts that found by Mengouo and colleagues in Cameroon [19]. The difference found in our study may be attributed to the higher population density experienced in most of the urban communities which aids transmission of rubella infection.

The role of sex in the distribution of cases is not well understood but our findings suggested more females were affected than males. This result is consistent with studies conducted in some parts of Nigeria, which shows that females had increased incidence of rubella than the males. For example, a study conducted in Jos, North Central Nigeria showed that 33% were males and 67% were females [20]. Similarly, Ume and Onye reported 41% rubella cases among males and 59% in females [21]. In Ethiopia, 54% of IgM positive cases were females higher than 46% reported among the males [18]. This may be because of the settings where more females are engaged in catering for children or the sick who might be exposed to the rubella infection. However the transmission of the disease is airborne and both sexes are equally at risk of the infection.

In this study majority of the rubella cases occurred in the children aged less than 15 years. This findings are similar to that by Mitiku, Bedada [18] that reported 94.7% of rubella positive cases in Ethiopia and Chimhuya, Manangazira [7] that also recorded 98% in Zimbabwe from this age group. Of particular interest is the adolescents’ females who might contract rubella during pregnancy and at the risk of giving birth to children with CRS. Therefore the inclusion of the rubella vaccine as part of the routine immunization can help to protect the entire population from rubella infection.

**Limitations:** the findings of this study are subjected to some limitations including; the case defintion for the detection of rubella cases which was designed for measles cases and may under report rubella cases, the existence of missing data on some variables which highlights some issues with data management, issues with pending laboratory results due to lack of reagents.

## Conclusion

Rubella affects children mostly less than 15 years. The rubella incidence was higher among females with majority of the cases occuring in the urban areas. There was a seasonal trend of the cases occurring during the dry season before the onset of the rainy season. With the introducton of the rubella vaccine the incidence of cases have declined significantly. However there is the need for the DSD in collaboration with WHO to develop a case definition to include all suspected cases of rubella. The surveillance or disease control officers should improve on data capture to prevent missing data. There is also the need for government to partner WHO to support the laboratory in confirming all suspected rubella cases especially in the elimination phase of the disease.

### What is known about this topic

- Rubella vaccine is known to be efficient cost-effective intervention for the control of rubella and its related complications (congenital rubella syndrome);
- It is also known that naive adolescent' females who might contract rubella during pregnancy risk for their babies developing CRS.

### What this study adds

- The study has systematically evaluated the current epidemiology of rubella in Ghana for the first time since the introduction of the rubella vaccine;
- There is significant reduction of the incidence of rubella cases in Ghana after the introduction of the rubella vaccine and could contribute to the elimination of the disease;
- There is the need for countries nearing elimination phase of rubella to redefined the case definition for rubella to include all cases.
